# Numerical Simulation to Predict COVID-19 Cases in Punjab

**DOI:** 10.1155/2022/7546393

**Published:** 2022-07-22

**Authors:** Vanshika Aggarwal, Geeta Arora, Homan Emadifar, Faraidun K. Hamasalh, Masoumeh Khademi

**Affiliations:** ^1^Department of Mathematics, School of Chemical Engineering and Physical Sciences, Lovely Professional University, India; ^2^Department of Mathematics, Hamedan Branch, Islamic Azad University, Hamedan, Iran; ^3^Department of Mathematics, College of Education, University of Sulaimani, Sulaimani, Kurdistan Region, Iraq

## Abstract

Coronavirus disease 2019 is a novel disease caused by a newly identified virus, Severe Acute Respiratory Syndrome Coronavirus 2 (SARS-CoV-2). India recorded its first case of COVID-19 on 30 January 2020. This work is an attempt to calculate the number of COVID-19 cases in Punjab by solving a partial differential equation using the modified cubic B-spline function and differential quadrature method. The real data of COVID-19 cases and Google Community Mobility Reports of Punjab districts were used to verify the numerical simulation of the model. The Google mobility data reflect the changes in social behavior in real time and therefore are an important factor in analyzing the spread of COVID-19 and the corresponding precautionary measures. To investigate the cross-border transmission of COVID-19 between the 23 districts of Punjab with an analysis of human activities as a factor, the 23 districts were divided into five regions. This paper is aimed at demonstrating the predictive ability of the model.

## 1. Introduction

SARS-CoV-2 was recognized as a new disease known as coronavirus disease 2019 (COVID-19) and was declared a pandemic by the WHO on March 11, 2020. In India, three cities in Kerala reported the first incident of COVID on January 30. The country was placed under total lockdown on March 25, 2020, which lasted until May 31, 2020. After that, the towns began to reopen gradually. Both infection rates and new and active patients began to decline in September. By January 2021, the number of daily cases had decreased to less than 15,000 from more than 90,000 in mid-September. The second wave, which began in March 2021, was far more devastating than the first. Regions of the country suffered shortages of vaccines, oxygen cylinders, hospital beds, and other medical supplies. By the end of April, India had surpassed the rest of the world in terms of new and active cases. On January 16, 2021, India began its vaccination program with the AstraZeneca vaccine (Covishield) and the indigenous Covaxin. Sputnik V and the Moderna vaccine were later licensed for emergency use as well. According to the CoWIN portal, India reached 100 crore (1 billion) vaccination doses on October 21, 2021, at 9:47 am [1].

A spatiotemporal PDE model is used in this work to forecast COVID-19 cases in Punjab, India. The model utilized the combined impact of the transboundary spread throughout Punjab regions with the impact of social distance effects. Many spatiotemporal models, such as [2–5], use PDEs to define infectious illnesses. This work is an attempt to predict COVID-19 cases using real-world data collected from the Google Community Mobility Reports. As locations provide real-time information about changes of population in their social behavior, mobility trends derived from location history are crucial to study COVID-19 spread and prevention.

There are some limitations with Google mobility data due to the dynamic nature of mobility patterns. One of the major reasons is that cell phones may not accurately reflect population mobility, especially in suburban areas where people are not using GPS technology [6].

This manuscript is divided into ten sections.  Section 1 briefly explains the problem. In Section 2, the data are explained using the PDE model in Section 3. Sections 4 and 4 briefly explain the differential quadrature method and the B-spline functions, with more details in Section 6. Sections 7 and 8 contain the prediction method and parameter estimation. Results are presented in Section 9, followed by concluding remarks in Section 10.

## 2. Description of the Data

In this work, the model is applied for the period July 1, 2020, to August 15, 2020. During this time, India was under unlock phases 2 and 3 when few places were reopened in a phased manner.

There are twenty-three districts in Punjab. Malerkotla is the 23^rd^ district of Punjab. The district was carved out of Sangrur district on 14 May 2021, but here, it has been taken as a part of Sangrur district as the data for Malerkotla district was not available separately. The twenty-two districts have been grouped into five regions as follows (Figure 1):

*(i) Region 1.* Pathankot, Gurdaspur, Amritsar, Tarn Taran, and Kapurthala.

*(ii) Region 2.* Hoshiarpur, Jalandhar, Shahid Bhagat Singh Nagar, and Rupnagar.

*(iii) Region 3.* Sahibzada Ajit Singh Nagar (Mohali), Patiala, Fatehgarh Sahib, and Ludhiana.

*(iv) Region 4.* Sangrur, Barnala, Mansa, and Bathinda.

*(v) Region 5.* Moga, Faridkot, Firozpur, Sri Muktsar Sahib, and Fazilka.

By summarizing the new COVID-19 cases from all districts in a region, the daily new cases of that region are calculated. Two time series of Google mobility reports have been created. The first category includes activities such as grocery stores and pharmacies, retail and recreational activities, workplaces and parks, and transit stops that are thought to increase COVID-19 cases; the second category of activities focuses on residential activities (activities at home) that may help prevent COVID-19 epidemics. The daily changes of each region are calculated by aggregating the changes of all counties within a region.

## 3. The PDE Model

The considered PDE model can be categorized as an internal/local process within each region and an external/global process. In the local process, people can become infected by social interactions with infected individuals within a region but can take steps to prevent COVID-19 from spreading, while in the global process, it is possible to become infected through social interactions with those who have been infected outside of a particular region. The considered five regions are embedded in a Euclidean space and mapped on the *x*-axis, with coordinates for the five regions [7]. The close arrangement of regions ensures a continuous model to study the spread of COVID-19 in the regions.

Let *C*(*x*, *t*) denote the COVID-19 cases in the Punjab region *x* at a particular time *t*. The model is defined as follows:

(1) $$\begin{array}{c} \left\{\begin{array}{c} \frac{\partial C\left(x,t\right)}{\partial t}=\frac{\partial }{\partial x}\left(d\left(x\right)\frac{\partial C\left(x,t\right)}{\partial x}\right)+r\left(t\right)l\left(x\right)a\left(x,t-14\right)C\left(x,t\right)-c\frac{h\left(x,t-14\right)C\left(x,t\right)}{k+C\left(x,t\right)},\\ C\left(x,t\right)=\psi \left(x\right),\;1<x<5,\\ \frac{\partial C\left(1,t\right)}{\partial x}=\frac{\partial C\left(5,t\right)}{\partial x}=0,\;\;t>1, \end{array}\right. \end{array}$$

where

(i) The term (*∂*/*∂x*)(*d*(*x*)(*∂C*(*x*, *t*)/*∂x*)) refers to the spread of COVID-19 cases across different regions of Punjab, where *d*(*x*) represents the rate at which COVID-19 spreads across different regions. This term has been commonly used in epidemiology [3, 8] to describe the geographical spread of infectious diseases. In this case, *d*(*x*) is assumed to be constant, which means that *d*(*x*) ≡ *d* > 0
(ii) *r*(*t*)*l*(*x*)*a*(*x*, *t* − 14)*C*(*x*, *t*) denotes new cases in a region *x* at time *t*, which is implemented frequently to discuss the growth of germs, cancers, and information over time [8]
  - The function *r*(*t*) > 0 represents the growth rate in COVID-19 cases at time *t* for all Punjab regions. Here, *r*(*t*) is assumed to increase with time *t* as the number of COVID-19 cases increases. Among the choices for representing the pattern, *r*(*t*) = *g*(*b*_1_ + *b*_2_*t*) and *g*(*u*) = 1/(1 + exp(−*u*)) have been chosen with the parameters *b*_1_ and *b*_2_, which are to be determined from COVID-19
  - The spatial diversity of COVID-19 is described by the location function *l*(*x*), which exhibits various infection rates in the five Punjab regions. The function *l*(*x*) can be created by using cubic spline interpolation in MATLAB. The gathered COVID-19 data is used to determine *l*(*x*)
  - *a*(*x*, *t* − 14) represents data taken from Google mobility reports for retail and recreation, groceries and pharmacies, parks and transit stations, and workplaces, all of which are expected to increase the number of COVID-19 cases. Because the effect of the activities may take up to two weeks, the PDE model time *t* is shortened by 14 days to account for the COVID-19 incubation period
(iii) The function *c*(*h*(*x*, *t* − 14)*C*(*x*, *t*)/(*k* + *C*(*x*, *t*))) shows a reduced rate of COVID-19 cases due to high precaution measures to limit contact. The Michaelis-Menten function was used to limit the impact of household activities on the spread of COVID-19
  - *h*(*x*, *t* − 14) describes the data of residential activities that help to prevent COVID-19 outbreaks, collected by Google mobility data, where *t* − 14 is the incubation period
  - Here, *c* denotes the maximum reduction rate for each region with the effect of government actions and personal precautions
  - *k* is the number of COVID-19 cases where the reduction rate is (1/2)*c*

*a*(*x*, *t* − 14) and *h*(*x*, *t* − 14) are obtained using Google mobility data, while the other constants *d*, *k*, and *c* and parameters of *r*(*t*) and *l*(*x*) are evaluated by the data of COVID-19 cases

*C*(*x*, 1) = *ψ*(*x*) is the initial function that describes the beginning states of COVID-19 in each region of Punjab and can be created by using cubic spline interpolation in MATLAB from the collected data of COVID-19 cases

To solve the PDE model, the boundary conditions are considered of Neumann type [8] given as

(2) $$\begin{array}{c} \frac{\partial C}{\partial x}\left(t,1\right)=\frac{\partial C}{\partial x}\left(t,5\right)=0,\;\;t>1. \end{array}$$

For simplicity, cases imported from neighboring states are counted as local Punjab cases, assuming that no COVID-19 spreads across the border when *x* = 1 and 5.

Many mathematical models have been used to discuss the mathematics intervention in the study of the spread of infectious diseases [9–11]. The classic models, namely, the susceptible, infectious, and recovered (SIR) model [12] and the susceptible, exposed, infectious, and recovered (SEIR) model [13], are the models generally used to study the spread and after-effects of COVID-19. Other proposed models are based on differential equations and statistical models [14, 15]. The present PDE model adopted in the study is based on the community model [7]. This model includes the impacts of personal precautions such as wearing face masks and maintaining social distance on COVID-19 cases at the district level. To the best of our knowledge, this work is the first attempt to apply PDE models on COVID-19 prediction with the Google Community Mobility Reports in Punjab, India.

## 4. Differential Quadrature Method

The differential quadrature method is a technique for approximating the derivatives of a function as a linear summation of function at the discrete knot points in the domain [16]. It was developed by the late Richard Bellman and his associates in the early 1970s. The following summation

(3) $$\begin{array}{c} u_{x}\left(x_{i}\right)=\overset{n}{\underset{j=1}{\sum }}a_{ij}u\left(x_{j}\right),\;\;i=1,2,\cdots ,n, \end{array}$$

is used to approximate the derivatives of function *u*(*x*) at any nodal point *x*_*i*_ of the partition. Here, *a*_*ij*_ are constant coefficients known as weighting coefficients which can be obtained in many ways.

The present work is intended to implement the B-spline basis functions of the third degree with modification in DQM to determine the weighting coefficients.

The idea of using the spline-based differential quadrature method to determine weighting coefficients was proposed by Bellman et al. [16], which was researched and improved by Quan and Chang [17, 18]. DQM has been implemented with various basis functions including the sinc functions, spline functions, and Lagrange interpolation polynomials [17, 18]. A lot of work has been reported in the literature for the advancement in the methodology for the selection of the grid points [19–21]. The Cubic B-spline has also shown accurate results for solving various PDEs using the DQM approach [22–26]. Third-order B-splines have advantages in terms of computational simplicity, numerical stability, and interpolated curve smoothness. Since both DQM and cubic B-spline functions have proven to be very effective, we chose to use this approach.

## 5. B-Spline

A spline of order *n* is a piecewise polynomial function of degree *n* − 1 in a variable *x*.

The values of *x* where the pieces of the polynomial meet are known as knots, denoted as *x*_0_, *x*_1_, *x*_2_, ⋯, *x*_*n*_, and sorted into nondecreasing order.

The third-degree B-spline called as the cubic B-spline basis function is given by the formula defined below with *h* as the knot span with the uniformly distributed knots, i.e., *h* = *x*_*i*+1_ − *x*_*i*_.

(4) $$\begin{array}{c} B_{\left(i,3\right)}\left(x\right)=\frac{1}{h^{3}}\left\{\begin{array}{cc} {\left(x-x_{i-2}\right)}^{3}, & x\in \left[x_{i-2},x_{i-1}\right),\\ {\left(x-x_{i-2}\right)}^{3}-4{\left(x-x_{i-1}\right)}^{3}, & x\in \left[x_{i-1},x_{i}\right),\\ {\left(x_{i+2}-x\right)}^{3}-4{\left(x_{i+1}-x\right)}^{3}, & x\in \left[x_{i},x_{i+1}\right),\\ {\left(x_{i+2}-x\right)}^{3}, & x\in \left[x_{i-2},x_{i-1}\right),\\ 0, & \text{otherwise}. \end{array}\right. \end{array}$$

From the definition, the values of *B*_*i*_(*x*) and its first and second derivatives at the nodal points can be tabulated.

The cubic B-spline basis functions are further implemented in the modified form to make the system diagonally dominant, defined as follows:

(5) $$\begin{array}{c} \left\{\begin{array}{c} M_{1}\left(x\right)=B_{1}\left(x\right)+2B_{0}\left(x\right),\\ M_{2}\left(x\right)=B_{2}\left(x\right)-B_{0}\left(x\right),\\ M_{i}\left(x\right)=B_{i}\left(x\right),\;\text{for }i=3,\cdots ,m-2,\\ M_{m-1}\left(x\right)=B_{m-1}\left(x\right)-B_{m+1}\left(x\right),\\ M_{m}\left(x\right)=B_{m}\left(x\right)+2B_{m+1}\left(x\right). \end{array}\right. \end{array}$$

Therefore, {*M*_1_, *M*_2_, ⋯, *M*_*m*_} now form a basis over the region.

## 6. Description of the Method

The first-order derivative approximation is given by

(6) $$\begin{array}{c} M_{p}^{\prime }\left(x_{i}\right)=\overset{m}{\underset{j=1}{\sum }}a_{ij}M_{p}\left(x_{j}\right),\;\text{for }i=1,2,\cdots ,m;p=1,2,\cdots ,m. \end{array}$$

Now, for the first knot point *x*_1_, that is, *i* = 1,

(7) $$\begin{array}{c} M_{p}^{\prime }\left(x_{1}\right)=\overset{m}{\underset{j=1}{\sum }}a_{1j}M_{p}\left(x_{j}\right),\;\text{for }p=1,2,\cdots ,m. \end{array}$$

For *p* = 1,

(8) $$\begin{array}{c} M_{1}^{\prime }\left(x_{1}\right)=a_{11}M_{1}\left(x_{1}\right)+a_{12}M_{1}\left(x_{2}\right)+a_{13}M_{1}\left(x_{3}\right)+\cdots +a_{1m}M_{1}\left(x_{m}\right),\\ B_{1}^{\prime }\left(x_{1}\right)+2B\prime_{0}\left(x_{1}\right)=a_{11}\left[B_{1}\left(x_{1}\right)+2B_{0}\left(x_{1}\right)\right]+a_{12}\left[B_{1}\left(x_{2}\right)+2B_{0}\left(x_{2}\right)\right]+a_{13}\left[B_{1}\left(x_{3}\right)+2B_{0}\left(x_{3}\right)\right]+\cdots ,\\ 0+\frac{-3}{h^{2}}=6a_{11}+1a_{12}+0a_{13}+0a_{14}+\cdots ,\\ \frac{-3}{h^{2}}=6a_{11}+1a_{12}+0+0+\cdots . \end{array}$$

Similarly, *p* = 2, 3, 4, ⋯, *m* provides equations in *m* variables. Thus, a system of *m* nonhomogenous equations in *m* variables is obtained with the matrix representation of the equations as follows:

(9) $$\begin{array}{c} \left[\begin{array}{ccccccc} 6 & 1 & 0 & \; & \; & \; & \;\\ 0 & 4 & 1 & 0 & \; & \; & \;\\ 0 & 4 & 4 & 1 & \; & \; & \;\\ \; & \ddots & \ddots & \ddots & \; & \; & \;\\ \; & \; & \; & 1 & 4 & 1 & 0\\ \; & \; & \; & 0 & 1 & 4 & 0\\ \; & \; & \; & \; & 0 & 1 & 6 \end{array}\right]\left[\begin{array}{c} a_{11}\\ a_{12}\\ a_{13}\\ \vdots \\ a_{1\left(m-1\right)}\\ a_{1m} \end{array}\right]=\left[\begin{array}{c} -\frac{6}{h}\\ \frac{6}{h}\\ 0\\ \vdots \\ 0\\ 0 \end{array}\right]. \end{array}$$

The “Thomas algorithm” is used to solve the above tridiagonal system of equations. The solution of which provides the coefficients *a*_11_, *a*_12_, ⋯, *a*_1*m*_.

Following the same process from *i* = 2 to *i* = *m* − 1, the value of coefficients *a*_*i*1_, *a*_*i*2_, ⋯, *a*_*im*_ is calculated. Hence, the weighing coefficients *a*_*ij*_ for *i* = 1, 2, ⋯, *m* and *j* = 1, 2, ⋯, *m* have been evaluated. Using these coefficients, the weighing coefficients *b*_*ij*_ for *i* = 1, 2, ⋯, *m* and *j* = 1, 2, ⋯, *m* are calculated by

(10) $$\begin{array}{c} b_{ij}=2a_{ij}\left(a_{ij}-\frac{1}{x_{i}-x_{j}}\right),\;\text{for }i\neq j,\\ b_{ii}=-\overset{m}{\underset{j=1,j\neq i}{\sum }}b_{ij}. \end{array}$$

## 7. Prediction Method

The implementation of the proposed scheme (DQM and modified cubic B-spline) turns the function derivative (*∂*/*∂x*)(*d*(*x*)(*∂C*(*x*, *t*)/*∂x*)) into a linear sum of function values at discrete points, which is further solved by the R-K approach using MATLAB. The values of the model parameters are to be determined by the collected data of COVID-19 cases in the five regions. In this work, the COVID-19 cases have been predicted one day ahead.

In order to predict COVID-19 cases, the parameters have first been trained and then the PDE is solved for prediction. The following algorithm explains the prediction procedure [7]:

- The data of the number of COVID-19 cases has been collected for the period July 1, 2020, to August 15, 2020. So there are a total of 46 days in this period
- The historical COVID-19 data for days 1-7 has been used to train the parameters for each region
- The fourth-order Runge-Kutta method is used in MATLAB to numerically solve the equation for prediction for day 8
- The collected data for days 2-8 is used to train the parameters and predict for day 9. This process is repeated till day 46 is predicted from the data collected for days 39-45
- The actual COVID-19 data for days 8-46 are then compared to the predicted data to check the accuracy

## 8. Estimated Parameters

The following are the values of the parameters used for the prediction of COVID-19 cases on the 8^th^, 9^th^, and 10^th^ days:

- *l*(*x*) represents the different infection rates of the five regions of Punjab. The daily infection rate is 7 days moving average of new cases per 100,000 residents
- As *r*(*t*) is the growth rate for all Punjab regions, therefore, *b*_1_ and *b*_2_ have only one value for each prediction step.  Table 1 shows the value of *l*_*i*_ for regions 1-5, respectively, and the constants *b*_1_ and *b*_2_
- *a*(*x*, *t* − 14) is a collection of data for retail and recreation, groceries and pharmacies, parks, transit stations, and workplaces from Google mobility data. The daily changes for each region were calculated by aggregating the changes of all counties within a region. The negative values of *a*(*x*, *t* − 14) reflect the decrease in mobility during this period compared to the baseline period
- The *h*(*x*, *t* − 14) entry represents the daily changes in residential activities of each region, which were calculated by aggregating the changes of all counties within a region. The positive values of *h*(*x*, *t* − 14) reflect an increase in time spent at home during this period compared to the baseline period
- *d* > 0 depicts how fast the infection spreads across different regions of Punjab. This has been calculated through the fminbnd function in MATLAB.  Table 2 represents the value of *a*(*x*, *t* − 14), *h*(*x*, *t* − 14), and *d* > 0 for the five regions
- The calculated values of *c* and *k* are shown in Table 3

## 9. Prediction Results and Accuracy

Figures 2–6 exhibit the predicted and actual COVID-19 cases in the five regions of Punjab from July 8, 2020, to August 15, 2020 (i.e., from day 8 to day 46). From the figures, we can see that for region 1 and region 2, the curve for the predicted and actual values intersects at many points, implying that the predicted value for that day is exactly the same as the actual value. For region 3, the curves do not intersect for more than one point and the predicted data has smaller values compared to the actual data, but both curves follow a similar pattern. For regions 4 and 5, the curves meet at few points and the predicted data has higher values than the actual data for the rest of the points. We can observe that for most of the points, the difference between both data is not huge and can be improved.

To analyze the model accuracy of prediction, the following formula has been used [7]:

(11) $$\begin{array}{c} 1-\left|\frac{x_{\text{real}}-x_{\text{predict}}}{x_{\text{real}}}\right|, \end{array}$$

where *x*_real_ represents the actual COVID-19 cases and *x*_predict_ represents the predicted COVID-19 cases. The accuracy for days 8, 9, and 10 for each region of Punjab is shown in Table 4.

The median of accuracy for regions 1-5 from day 8 to day 46 is 63.79%, 59.45%, 46.22%, 14.55%, and -10.91%, respectively. The accuracy achieved is relatively low, which could be due to certain limitations of this model as it does not include recovered cases. A person who has recovered from COVID-19 has low chances of being infected again, which affects the rate of infection. Google mobility reports also have certain limitations. As Punjab has many rural areas where GPS-enabled smartphones are not widely used, this affects the reliability of Google mobility data.

## 10. Conclusion

This work is an attempt to analyze the effectiveness of a partial differential equation model to predict the number of COVID-19 cases in Punjab, India. For this, 23 districts of Punjab were distributed into 5 groups/regions. The real-time data of COVID-19 as well as the Google mobility reports have been used for the calculation. The differential quadrature method and modified cubic B-spline functions have been used to convert the PDE into an ordinary differential equation, which has been further solved using the fourth-order Runge-Kutta method. All the numerical simulations have been performed using MATLAB. The actual COVID-19 data and the predicted data for regions 1-5 have been compared. From Figures 2–6, it can be seen that for many points, the model gives predicted values exactly the same as the actual data. The accuracy of the model for regions 1-5 from day 8 to day 46 is 63.79%, 59.45%, 46.22%, 14.55%, and -10.91%, respectively. The PDE model and the techniques used are found to be effective. A lot of work done has been proposed by researchers to analyze the spread of COVID-19 using an ordinary differential equation model, but a PDE model is rare. Keeping certain limitations of this model into consideration, this work shows the effectiveness of the PDE model, which has been found to be a suitable model which can be further optimized with the additional conditions.

## Figures and Tables

**Figure 1:** Punjab region-wise map.

**Figure 2:** Region 1.

**Figure 3:** Region 2.

**Figure 4:** Region 3.

**Figure 5:** Region 4.

**Figure 6:** Region 5.

**Table 1:** Values of *l*(*x*) and *b*_1_ and *b*_2_ for each region.

Day	*l*_1_	*l*_2_	*l*_3_	*l*_4_	*l*_5_	*b*_1_	*b*_2_
8	0.00024	0.00036	0.00075	0.000204	0.00016	-1.12989855522384	0.486179328647
9	0.00023	0.000456	0.00071	0.000207	0.00017	0.23123746155289	0.223507765687
10	0.00026	0.000489	0.00079	0.00022	0.000163	0.05590503704454	0.182044663455

**Table 2:** Values of *a*(*x*, *t* − 14), *h*(*x*, *t* − 14), and *d* for each region.

Day	*a*_1_	*a*_2_	*a*_3_	*a*_4_	*a*_5_	*h*_1_	*h*_2_	*h*_3_	*h*_4_	*h*_5_	*d*
8	-7.55	-5.33	-7.51	-5.07	-6.52	0.36	0.37	0.4	0.28	0.35	1.00006242294666
9	-8.46	-5.77	-7.67	-5.19	-6.57	0.46	0.38	0.44	0.27	0.39	1.00006242294666
10	-8.73	-5.7	-7.68	-5.77	-7.89	0.48	0.4	0.44	0.31	0.49	2.50032339920933

**Table 3:** Values of *c* and *k* for each region.

Day	*c*_1_	*c*_2_	*c*_3_	*c*_4_	*c*_5_

8	0.86615517325	0.80627260171	0.55263705137	0.91398293398	0.91252678272
9	0.86598826807	0.79387503186	0.66494079048	0.85666148707	0.90812006030
10	0.84562520870	0.79627529187	0.64560647659	0.85195319277	0.90812006030

Day	*k*_1_	*k*_2_	*k*_3_	*k*_4_	*k*_5_

8	-1.49844358466	-1.54661440808	-18.40068405369	-0.27581339704	-0.54914780383
9	-1.51076173533	-1.61352531942	-7.56569956492	-1.41305273105	-0.57845985242
10	-2.01162262530	-1.46907399870	-7.84865807934	-1.59337848008	-0.57845985242

**Table 4:** Accuracy for regions 1, 2, 3, 4, and 5.

Day	1	2	3	4	5
8	5.0254%	56.4400%	5.0254%	-157.4534%	35.0215%
9	43.472%	38.297%	14.109%	80.424%	80.424%
10	60%	59.452%	51.058%	-17%	-342.5%

## Data Availability

The data used for the analysis of the model is available on http://www.google.com/covid19/mobility/. COVID-19 data for daily new cases can be found at https://www.covid19india.org/state/PB and https://www.mohfw.gov.in/.

## Abbreviations

PDE: Partial differential equation
GPS: Global Positioning System
DQM: Differential quadrature method.
